This article has been retracted.

# Niches of nine mangrove species in a *Sonneratia apetala*‐colonized area of Dongzhai Harbor, Hainan Island, China

**DOI:** 10.1002/ece3.6823

**Published:** 2020-10-04

**Authors:** Feng Wu, Baowen Liao, Yujun Chen, Zhongmao Jiang, Yunpeng Guo, Mei Li

**Affiliations:** ^1^ Key Laboratory of State Forestry Administration on Tropical Forestry Research Research Institute of Tropical Forestry Chinese Academy of Forestry Guangzhou China; ^2^ Zhaoqing Xinghu National Wetland Park Management Center Zhaoqing China

**Keywords:** Dongzhai Harbor, Hainan Island, mangrove plant species, niche breadth, niche overlap, *Sonneratia apetala* diffusion area

## Abstract

The distribution of mangroves is influenced by the environment. We aimed to understand the ecological adaptability of various mangrove species within the range of the exotic species, *Sonneratia apetala* Buch.‐Ham., in Dongzhai Harbor, Hainan Island, China. We used three niche breadth indexes (Simpson, Levins, and Shannon–Weiner) and two niche overlap indexes (Pianka and Levins) to quantitatively determine the niche characteristics of nine mangrove species. The results showed that the order of the niche breadth values of mangrove species was as follows: *Aegiceras corniculatum* (Linn.) Blanco > *Kandelia obovata* Sheue et al. > *Bruguiera gymnorrhiza* (L.) Poir. > *Avicennia marina* (Forsk.) Vierh. Hailanci > *S. apetala* > *S. caseolaris* (L.) Engl. > *Rhizophora stylos*a Griff > *Ceriops tagal* (Perr.) C. B. Rob. > *B. sexangula* (Lour.) Poir. Pearson correlation analysis revealed that the niche breadth of each population was significantly correlated with the importance value of the population in the whole sample (R_1_ = R_2_ = 0.771, R_3_ = 0.644, *p* < .05). The nine mangrove species were divided into three groups by Bray–Curtis cluster analysis; the groups were similar to the distribution of mangrove species in the natural state as determined by tide level. Niche similarity analysis showed that the niche similarity of most mangroves ranged between 0.5 and 0.8 and that the species pairs *A. corniculatum*–*B. gymnorrhiza*, *A. corniculatum*–*Avicennia marina,* and *K. obovata–S. caseolaris* were characterized by large niche similarity ratios. Although it had a moderate niche breadth, *S. apetala* had a relatively broad niche overlap with mangroves in the mid‐ and low‐tide zones (*S. caseolaris*, *A. corniculatum*, *K. obovata*, and *Avicennia marina*), a moderate overlap with *B. gymnorrhiza* and *R. stylosa*, only a slight overlap with *C. tagal*, and no overlap with *B. sexangular*. There was no obvious linear relationship between niche width and niche overlap of mangroves. Due to its inefficiency in utilizing certain resources and relatively high degree of resource selection, it seems likely that *S. apetala* will not pose a threat to the survival of native plants, let alone completely replace native species.

## Graphical abstract

Experts have different opinions on whether *Sonneratia apetala* is defined as an invasive species. In this paper, we investigated the growth and succession of *S. apetala*, which was introduced to China for many years to determine whether the *S. apetala* would pose a threat to the survival of the local species according the niche theory. The results obtained in this study will provide a theoretical basis for further elucidating the interspecific relationships among exotic and native mangrove species and for the rational utilization of *S. apetala*.

## 1 INTRODUCTION

The study of the species niche is an important area of modern ecological theory. The niche concept was first proposed by Grinnell (1917) in the early 20th century. At present, there are still considerable differences in opinion regarding the concept, calculation method (Aguiar‐Melo et al., 2019; Anderson, 2013), and interpretation of the niche. However, the theory is still used by scientists to solve practical problems. Numerous studies have been conducted using niche theory (Ingram et al., 2018; Winemiller et al., 2015), measurement (Bai et al., 2018; Gaston & Speicer, 2001), application, and practice (López‐Alvarez et al., 2015; Mutshida & O'Hara, 2011). Niche theory has played an important role in the study of community species composition, structure and function, inter‐species relationship, biodiversity (Zuppinger‐Dingley et al., 2014), community dynamic succession, and population evolution (Lou et al., 2018; Sullivan et al., 2018).

An important aspect of niche theory is the quantitative measurement of niche breadth (or niche width), niche similarity, and niche overlap (Du et al., 1997; Su et al., 2003). These aspects have been used in numerous niche‐based studies on different vegetation types and populations (Aiba et al., 2012; Arellano et al., 2014), including forest vegetation (Liu et al., 2018; Marinšek et al., 2015), desert vegetation (Chen et al., 2019), wetland vegetation (Alleman & Hester, 2011; Rojo et al., 2016), rare and endangered species (Adhikari et al., 2019; Iannella et al., 2018; Mays et al., 2018), microorganisms (Dann et al., 2019; Li et al., 2019; Trivedi et al., 2019), insects (Rodgers et al., 2019), and birds (Pagani‐Núñez et al., 2019). As a species that was introduced to China and planted in large numbers in the coastal areas of south China, *Sonneratia apetala* Buch.‐Ham inevitably occupies a certain ecological niche and competes for essential resources with native tree species, even potentially threatening the survival of native mangroves (Ren et al., 2007). This leads to the question: will *S. apetala* monopolize the ecological resources and be the only survivor in a long biological succession resulting in the extinction of native mangroves?

In this study, we employed a quantitative ecology approach to examine the niche breadth, niche similarity, and niche overlap of mangrove species in the diffusion zone of the exotic mangrove, *S. apetala,* in Dongzhai Harbor, Hainan Island, China. We anticipate that the results from this study will provide a theoretical basis for further elucidating the interspecific relationships among exotic and native mangrove species and for the rational utilization of *S. apetala*.

## 2 METHODS

The study site is located in the Dongzhai Harbor mangrove area (110°32ʹ–110°37ʹE, 19°51ʹ–20°01ʹN) in the northeastern region of Hainan Island, China. The area experiences a tropical monsoon marine climate, with an annual average temperature of 23.3–23.8°C, a maximum temperature of 38.9°C, a minimum temperature of 2.6°C, and an annual average of more than 20:00 hr of sunshine. The annual average relative humidity is 85%, and annual average precipitation is 1,676.4 mm. The rainy season typically commences in the first 10 days of May and ends during the second 10 days of October. The tidal pattern in the coastal areas is irregular and semi‐diurnal, with a maximum tidal range of 1.8 m and a mean tidal range of 1.1 m. The wide intertidal zone provides an extensive area for mangrove growth.

Mangroves in the Dongzhai Harbor Mangrove Area cover an area of 2,006 ha and comprises 26 native mangrove species belonging to 16 genera within 13 families, along with 1 introduced species (*S. apetala*). *S. apetala* was introduced to Dongzhai Harbor from Bangladesh in 1985, and after 3 years, it had become well established. The maximum tree height recorded in 2003 was 13.5 m (Liao et al., 2003). At present, *S. apetal* had been planted over 3,800 ha in China, accounting for 10.5% of the total mangrove area in China (Jiang et al., 2019).

### 2.1 Sample plots survey

The experimental plots used in this study were located in the Sanjiang Mangrove Area of Dongzhai Harbor Nature Reserve (the area of mangroves here is approximately 1,000 ha). In 1989, approximately 1 ha of *S. apetala* plantation was located in this forest area and by 1996, the area of *S. apetala* plantation had increased to approximately 10 ha. *S. apetala* dispersed primarily upstream and downstream along both sides of the Yanzhou and Meipo rivers. The range of *S. apetala* dispersal and colonization has occurred within an area characterized by a successional series of *Kandelia obovata* Sheue et al. + *Aegiceras corniculatum* (Linn.) Blanco communities. The successional community types in this area and their substitution order are as follows: *K. obovata* + *A. corniculatum* (Community I) → *A. corniculatum* + *K. obovata* (Community II) → *A. corniculatum* + *K. obovata* + *Bruguiera gymnorrhiza* (L.) Poir. (community III) → *A. corniculatum* + *B. gymnorrhiza* + *K. obovata* (community IV).

The experimental plots (measuring 10 m × 10 m) were all located within these communities, among which 32, 10, 10, and 14 plots were established in communities I, II, III, and IV, respectively. Mangroves in the quadrat that were over 2 cm of ground diameter were measured and the name of species, number of individuals per species, coverage, diameter at breast height (DBH), and tree height were recorded. Although small numbers of *Acanthus illicifolius* L. and *A. illicifolius* var. *ebracteatus* (Vahl) Williams were also distributed in each community, these were not included in data collection owing to their small size and low numbers.

### 2.2 Statistical analysis

#### 2.2.1 Species importance values

Relative importance values can accurately reflect the utilization efficiency of environmental resources by tree species and negate differences relating to individual size. Accordingly, we used relative importance values instead of relative individual proportion numbers when measuring niche width and niche overlap, based on relative density (RD), relative frequency (RF), and relative significance (RS). In this study, the importance value was used as a measurement index of the dominant species and was determined using the following equation:

$$\text{IV}\;=\;\left(\text{RD + RF + RS}\right)÷3$$

RD = number of a certain plant species/ number of all plant species × 100%

RF = frequency of a certain plant species/ frequency of all plant species × 100%

RS = sum of DBH square of a certain plant species/ sum of DBH square of all plant species × 100%

Where IV is the importance value (Song, 2001), RD is the relative density, RF is the relative frequency, and RS is the relative significance (Liu et al., 2018).

#### 2.2.2 Niche breadth

We used the following formulae to assess niche breadth:

Simpson formula: $B_{i1}=1/\left(\sum_{j=1}^{r}P_{\mathrm{ij}}^{2}\right)\;\left(1\right)$ (Simpson, 1949)

Levins formula: $B_{i2}=1/\left(r\sum_{j=1}^{r}P_{\mathrm{ij}}^{2}\right)\;\left(2\right)$ (Levins, 1968）

Shannon–Wiener formula: $B_{i3}=‐\sum_{j=1}^{r}P_{\mathrm{ij}}\ln P_{\mathrm{ij}}\;\left(3\right)$ (Hu et al., 2009; Shannon & Weiner, 1949).

In these formulae, *B_i_*_1,_ *B_i_*_2_, and *B_i_*_3_ are species niche breadths. *P_ij_* is the proportion of IV of species *i* in the community *j*, and *r* is the number of communities.

#### 2.2.3 Niche similarity

Schoener formula: $C_{\mathrm{ik}}=1‐1/2\sum_{j=1}^{r}\left|P_{\mathrm{ij}}‐P_{\mathrm{kj}}\right|\;\left(4\right)$ （Schoener, 1968; Hurlbert, 1978）

In this formula, *C_ik_* is the niche similarity of species *i* and species *k*, *C_ik_* = *C_ki_*, with range (0, 1); *P_ij_* and *P_kj_* are the proportion of IV of species *i* and species *k* in the community *j*, and *r* is the number of communities.

#### 2.2.4 Niche overlap

Pianka formula: $O_{\mathrm{ik}}^{\prime }=\sum_{j=1}^{r}P_{\mathrm{ij}}P_{\mathrm{kj}}/\sqrt{\sum_{j=1}^{r}P_{\mathrm{ij}}^{2}\sum_{j=1}^{r}P_{\mathrm{kj}}^{2}}\;\left(5\right)$ (Pianka, 1973)

Levins formula: $O_{\mathrm{ik}}^{\prime }=B_{i2}\sum_{j=1}^{r}P_{\mathrm{ij}}P_{\mathrm{kj}}\;\left(6\right)$ (Levins, 1968)

In these formulae, $O_{\mathrm{ik}}^{\prime }$ and $O_{\mathrm{ik}}^{\prime \prime }$ are the niche overlap values of species *i* to species *k*. *B_i_*_2_ is the niche breadth of species; thus $O_{\mathrm{ik}}^{\prime }\neq O_{\mathrm{ik}}^{\prime \prime }$.

We used Excel 2016 and R 3.4.3 (Lucent Technologies, New Jersey, USA.) for calculating the importance values and niche characteristics, respectively. PAST v3.10 (Øyvind Hammer, Natural History Museum, University of Oslo, Norway) was used for Bray–Curtis clustering of species by niche width (Gong & Lv, 2017), and produced the cluster result graph (Figure 3). Origin 2018 (OriginLab, Northampton, Massachusetts, USA) was used to generate figures (Figures 1, 2 and 4, 5, 6).

**FIGURE 1:** Importance values of different mangrove species in the extension area of *S. apetala*

**FIGURE 2:** Niche breadth values for different mangrove species in the extension area of *S. apetala*

## 3 RESULTS

### 3.1 Importance value characteristics of mangroves

Among the 66 sample plots, we recorded the presence of nine species, from seven genera within five families. As shown in Figure 1, the order of the average importance value of mangrove species was as follows: *A. corniculatum* (41.07 ± 9.81) > *K. obovata* (25.86 ± 13.25) > *B. gymnorrhiza* (13.85 ± 7.25) > *Avicennia marina* (Forsk.) Vierh. Hailanci (6.73 ± 4.19) > *S. apetala* (4.79 ± 3.38) > *S. caseolaris* (L.) Engl. (4.59 ± 3.94) > *Rhizophora stylos*a Griff (1.42 ± 1.91) > *Ceriops tagal* (Perr.) C. B. Rob. (1.08 ± 1.34) > *B. sexangula* (Lour.) Poir. (0.63 ± 1.26).

### 3.2 Niche breadth

As shown in Figure 2, the niche breadth values obtained using the formulae (1), (2), and (3) are somewhat different. However, regardless of the formula used, the order of the calculated niche breadth values was the same, as follows: *A. corniculatum* > *K. obovata* > *B. gymnorrhiza* > *Avicennia marina* > *S. apetala* > *S. caseolaris* > *C. tagal* > *R. stylosa* > *B. sexangula*. This is consistent with the order of the average importance value of the population in the whole sample. Pearson correlation analysis revealed that the niche width of each population was significantly correlated with the importance value of the population in the whole sample (R_1_ = R_2_ = 0.771, R_3_ = 0.644, *p < *.05).

In order to explore the overall characteristics and similarities of niche breadth among species, the clustering analysis of species niche breadth was conducted by Bray–Curtis similarity index. Species are clustered according to the length of the Bray‐Curtis distance. The close species get together first, and those that are far away get together again. Our Bray–Curtis cluster analysis divided the mangrove community species into three groups (Figure 3), among which group 1 contained only *B. sexangula* with the lowest niche width, group 2 contained *R. stylosa* and *C. tagal*, and group 3 included the remaining six species. All species in group 3 were characterized by a large niche width. Of the nine mangrove species, *B. sexangula* was distributed at the high‐tide level, *R. stylosa* and *C. tagal* were distributed at the mid‐ to high‐tide level, and the remaining species were distributed at the mid‐ or low‐tide level. We discovered that the distribution results obtained using Bray–Curtis clustering closely mirrored the natural distribution of mangroves, thereby indicating that this classification can be used objectively to characterize the adaptability of mangroves to the tide level.

**FIGURE 3:** Bray–Curtis similarity clustering analysis of the niche breadth of mangrove trees

### 3.3 Niche similarity

As shown in Table 1, the niche similarity ratio of mangrove species is relatively high, with most lying between 0.5 and 0.8. The species pairs with the largest niche similarity were *A. corniculatum*–*B. gymnorrhiza, A. corniculatum–Avicennia marina,* and *K. obovata–S. caseolaris,* whereas those pairs with the lowest niche similarity were *S. apetala*–*B. sexangula*, *R. stylosa*–*B. sexangula,* and *S. caseolaris–B. sexangula*. The nine species recorded in the 66 sample plots formed a total of 36 species pair relationships, for which the niche similarity ratios were as follows (Figure 4). The ratios with the most pairs were 0.7–0.8, 0.6–0.7 and 0.5–0.6 with 6, 6 and 7 pairs, respectively. No pairs were found in the ratio ranges 0.9–1.0 and 0.1–0.2.

**TABLE 1:** Niche similarity of plant populations in the tree layer of the mangrove community

Species	A	B	C	D	E	F	G	H	I
A	1	0.7529	0.6657	0.5608	0.5694	0.5503	0.8064	0	0.3588
B		1	0.739	0.8079	0.7896	0.5434	0.6507	0.2471	0.5676
C			1	0.7021	0.6614	0.3354	0.7711	0.2289	0.3775
D				1	0.7467	0.423	0.5608	0.4392	0.6475
E					1	0.674	0.5638	0.2271	0.4331
F						1	0.476	0	0.2857
G							1	0	0.217
H								1	0.6412
I									1

Abbreviations: A, *S. apetala*; B, *A. corniculatum*; C, *K. obovata*; D, *B. gymnorrhiza*; E, *A. marina*; F, *R. stylosa*; G, *S. caseolaris*; H, *B. sexangula*; I, *C. tagal*.

**FIGURE 4:** Distribution map of the ecological niche similarity of mangrove trees. Each line represents a certain niche similarity coefficient range. The blue dot represents the numbers of species within a niche similarity.

### 3.4 Niche overlap

As shown in Figures 5 and 6, the amount of niche overlap between two similar species varied, but the trend was the same. The Pianka formula is simple and symmetrical, and it can reflect the overlap of species in relation to resource utilization. In a study examining the seaward ecological species of mangroves, Lin considered that the Pianka formula would be particularly applicable in reflecting the differences of mangrove species in resource utilization (Lin, 1997). As shown in Figure 5, the niche overlap between different species varies greatly (0–0.91). The niche overlap value of *S. caseolaris* and *K. obovata* was the highest (0.91), while the niche overlap value of *S. apetala* and *B. sexangula* was the lowest (0). In addition, we found that the niche overlap of two species in the same group was often greater than that of two species in different groups.

**FIGURE 5:** Niche overlap values for different mangrove species (Pianka values). The colors from blue to red indicate the degree of niche overlap (0–1.0). The number in the square where the two species meet indicates the value of niche overlap.

**FIGURE 6:** Niche overlap values for different mangrove species (Levins values)

## 4 DISCUSSION

1. Niche breadth is defined as the range of environmental conditions and resources that a species can utilize and it can vary from very broad (i.e., generalist species) to very narrow (i.e., specialist species) (Dantas et al., 2017; Dawson & Ellis, 1996). In the *S. apetala* diffusion area in Dongzhai Harbor, the niche breadth sizes of the nine recorded tree species could be ordered as *A. corniculatum* > *K. obovata* > *B. gymnorrhiza* > *Avicennia marina* > *S. apetala* > *S. caseolaris* > *C. tagal* > *R. stylosa* > *B. sexangula*, which provides a good reflection of the ecological adaptability and resource utilization capacity of these mangrove tree species. The niche breadth of *A. corniculatum*, *K. obovata*, *B. gymnorrhiza*, and *Avicennia marina* was higher than that of the other species examined (Figure 2). These results indicate that the aforementioned four species have the most abundant resources for growth and use, and a strong ability to utilize the available resource spectrum.

The niche breadth value (*B_i_*_1_ = 2.91) of *S. apetala* falls within an intermediate level, which is lower than that of the aforementioned four mangrove species (*B_i_*_1_ = 3.10–3.84), but higher than that of *S. caseolaris*, *C. tagal*, *R. stylosa*, and *B. sexangula*. This indicates that although *S. apetala* is a pioneer mangrove tree species that colonizes the frontier shore zone, its natural dispersal may be restricted by multiple factors. First, the optimum salinity level for the germination of *S. apetala* seeds is <5‰, and when the salinity is higher than 10‰, seed germination is inhibited and the tender buds of seedlings can show evidence of necrosis and rot due to salt injury (Wang et al., 1995). Second, the fruit of *S. apetala* generally matures in autumn. When temperatures fall below 5°C, naturally established seedlings can succumb to low‐temperature injuries and fail to overwinter. Third, the seedlings of *S. apetala* are heliophilic and are unable to grow and regenerate under the shade of dense canopies, and accordingly, this species does not readily invade closed virgin mangrove forests. In addition, the seeds of *S. apetala* are often consumed by birds and crabs (Zhang, 1995); thus, the seed germination rate tends to be low under natural conditions. These factors contribute to limiting the niche breadth of *S. apetala*. However, unlike the congeneric species, *S. caseolaris*, it has adapted to growing in habitats in which the temperature can fall to as low as 3°C. The naturally colonizing seedlings of *S. apetala* are not as susceptible as *S. caseolaris* to low temperatures in winter; thus, the calculated niche breadth of *S. apetala* is slightly larger than that of *S. caseolaris*.

2. The Bray–Curtis cluster analysis performed in this study divides the mangrove species of the different communities into three groups. The first of these groups contains a single species with a narrow niche width, indicating that this plant is a specialist with an extremely uneven distribution. The second group contains two species, with wider ecological niches, stronger resource utilization, and higher environmental adaptability. The third group contains species with the widest niches and distribution. These species tend to be generalists that can grow well in their respective habitats and play an important role in community level establishment.

3. Niche overlap reflects the utilization of the same habitat by two or more species and the spatial configuration among species. It is also indicative of the degree of similarity and competition among species with respect to resource utilization (Abrams, 1980; Spies et al., 1990). It is generally believed that niche overlap is closely related to niche width. For example, in this study, we discovered that the highest niche overlap (0.91) occurred between two species with large niche widths. Conversely, there appears to be little or no overlap between species with smaller niche widths (Dong et al., 2019; Lou et al., 2018; Walker, 1995), as exemplified in this study by *R. stylosa* and *C. tagal*, which have small niche breadths and the lowest niche overlap (0.18). Nevertheless, related research has indicated that the niche overlap between species is also associated with the ecological habits of species, with some species characterized by small niche breadth, but with similar ecological habits, potentially showing high niche overlap. Similarly, those species with high niche breadth, but different biological ecological habits, may appear to have low niche overlap due to contrasting resource usage (Lin, 1997). The results obtained in this study tended to be consistent with these assumptions. For example, we observed that *S. apetala* and *S. caseolaris*, with intermediate niche widths, had a high niche overlap value (0.90). Our results tended to emphasize the fact that there were no prominent patterns regarding the relationships between the niche width and niche overlap of mangroves in the Dongzhai Harbor mangrove community, thereby implying that the relationships between species are likely to be complex. This is consistent with the findings of previous studies (Aguiar et al., 2013; Lanszki et al., 2019; Martínez, 2010; Sá‐oliveira et al., 2014).

## 5 CONCLUSIONS

As an exotic introduced species, the niche of *S. apetala* in the mangrove community deserves close attention. The results of our niche breadth calculations revealed that the niche breadth of *S. apetala* was of an intermediate value, being lower than that of native mangroves in the mid‐ to low‐tidal flat zone (i.e., *A. corniculatum*, *K. obovata*, *Avicennia marina,* and *B. gymnorrhiza*), higher than that of native mangroves in the mid‐ to high‐tidal flat zone (i.e., *C. tagal*, *R. stylosa*, and *B. sexangula*), and similar to that of the congeneric species *S. caseolaris*. Niche overlap determinations indicated that the niche overlap between *S. apetala* and native mangroves in the mid‐ to low‐tidal flat zone (i.e., *S. caseolaris*, *A. corniculatum*, *K. obovata,* and *Avicennia marina*) was relatively large, whereas the overlap between *S. apetala* and native mangroves in the mid‐ to high‐tidal flat zone (*C. tagal*, *R. stylosa*, and *B. sexangula*) was relatively small. Accordingly, under conditions of resource insufficiency, it might be predicted that there would be strong competition for resources between *S. apetala* and native mangroves in the mid‐ to low‐tidal flat zone. However, owing to its inefficiency in utilizing certain resources and a relatively high degree of resource selection, it seems unlikely that *S. apetala* would completely replace those mangroves with which it has a high degree of niche overlap. Similarly, given the assumed weak competition between *S. apetala* and native mangroves in the mid‐ to high‐tidal flat zone, the probability of this alien species supplanting these native species also appears to be relatively low. Indeed, on the intertidal flats where it occurs, *S. apetala* tends to grow primarily in regions adjacent to rivers with a higher freshwater influx and deep silt. With the silting up of shores and the closure of the tree canopy, mangrove forest habitats may become increasingly unsuitable for the growth of *S. apetala*. Therefore, from the perspective of niche theory, we predict that this alien species will not pose a threat to the survival of native plants, let alone completely replace native species.

## CONFLICTS OF INTEREST

The authors declare no conflict of interest.

## AUTHOR CONTRIBUTION

**Feng Wu:** Formal analysis (equal); Software (lead); Writing‐original draft (lead); Writing‐review & editing (lead). **Baowen Liao:** Conceptualization (equal); Supervision (lead). **Yujun Chen:** Investigation (equal); Methodology (equal). **Zhongmao Jiang:** Investigation (equal); Methodology (equal). **Yunpeng Guo:** Formal analysis (equal); Investigation (equal). **Mei Li:** Conceptualization (equal); Funding acquisition (lead); Resources (lead).

## Data Availability

The raw data are available at Dryad with this https://doi.org/10.5061/dryad.qv9s4mwcc.

## References

[ece36823-bib-0001] Abrams, P. (1980). Some comments on measuring niche overlap. Ecology, 61(1), 44–49. 10.2307/1937153

[ece36823-bib-0002] Adhikari, D. , Tiwary, R. , Singh, P. P. , Upadhaya, K. , Singh, B. , Haridasan, K. E. , Bhatt, B. B. , Chettri, A. , & Barik, S. K. (2019). Ecological niche modeling as a cumulative environmental impact assessment tool for biodiversity assessment and conservation planning: A case study of critically endangered plant *Lagerstroemia minuticarpa* in the Indian Eastern Himalaya. Journal of Environmental Management, 243, 299–307. 10.1016/j.jenvman.2019.05.036 31102897

[ece36823-bib-0003] Aguiar, C. M. L. , Santos, G. M. , De, M. , Martins, C. F. , & Presley, S. J. (2013). Trophic niche breadth and niche overlap in a guild of flower‐visiting bees in a Brazilian dry forest. Apidologie, 44(2), 153–162. 10.1007/s13592-012-0167-4

[ece36823-bib-0004] Aguiar‐Melo, C. , Zanella, C. M. , Goetze, M. , Palma‐Silva, C. , Hirsch, L. D. , Neves, B. , Costa, A. F. , & Bered, F. (2019). Ecological niche modeling and a lack of phylogeographic structure in *Vriesea incurvata* suggest historically stable areas in the southern Atlantic Forest: Phylogeography of *Vriesea incurvata* . American Journal of Botany, 106(7), 971–983. 10.1002/ajb2.1317 31247130

[ece36823-bib-0005] Aiba, M. , Takafumi, H. , & Hiura, T. (2012). Interspecific differences in determinants of plant species distribution and the relationships with functional traits. Journal of Ecology, 100(4), 950–957. 10.1111/j.1365-2745.2012.01959.x

[ece36823-bib-0006] Alleman, L. K. , & Hester, M. W. (2011). Refinement of the fundamental niche of black mangrove (*Avicennia germinans*) seedlings in Louisiana: Applications for restoration. Wetlands Ecology and Management, 19(1), 47–60. 10.1007/s11273-010-9199-6

[ece36823-bib-0007] Anderson, R. P. (2013). A framework for using niche models to estimate impacts of climate change on species distributions. Annals of the New York Academy of Sciences, 1297(1), 8–28. 10.1111/nyas.12264 25098379

[ece36823-bib-0008] Arellano, G. , Cala, V. , & Macía, M. J. (2014). Niche breadth of oligarchic species in Amazonian and Andean rain forests. Journal of Vegetation Science, 25(6), 1355–1366. 10.1111/jvs.12180

[ece36823-bib-0009] Bai, H. H. , Wang, X. F. , & Xu, J. G. (2018). Nutrition ecological niche of dominant arbor species in natural *Pinus taiwanensis* community. Journal of Nanjing Forestry University(Natural Science Edition), 42(2), 81–88. 10.3969/j.issn.1000-2006.201706043

[ece36823-bib-0010] Chen, L. , Xin, J. N. , Su, Y. , Li, Y. F. , Song, N. P. , Wang, L. , Yang, X. G. , & Bian, Y. Y. (2019). Effects of heterogeneous habitats on community composition and niche characteristics of different plant populations in the deserts steppe of China. Acta Ecologica Sinica, 39, 1–19.

[ece36823-bib-0011] Dann, L. M. , Clanahan, M. , Paterson, J. S. , & Mitchell, J. G. (2019). Distinct niche partitioning of marine and freshwater microbes during colonisation. FEMS Microbiology Ecology, 95(8), 10.1093/femsec/fiz098 31271413

[ece36823-bib-0012] Dantas, M. A. T. , Cherkinsky, A. , Bocherens, H. , Drefahl, M. , Bernardes, C. , & França, L. D. M. (2017). Isotopic paleoecology of the Pleistocene megamammals from the Brazilian Intertropical Region: Feeding ecology (δ13C), niche breadth and overlap. Quaternary Science Reviews, 170, 152–163. 10.1016/j.quascirev.2017.06.030

[ece36823-bib-0013] Dawson, T. J. , & Ellis, B. A. (1996). Diets of mammalian herbivores in Australian arid, hilly shrublands: Seasonal effects on overlap between euros (hill kangaroos), sheep and feral goats, and on dietary niche breadths and electivities. Journal of Arid Environments, 34(4), 491–506. 10.1006/jare.1996.0127

[ece36823-bib-0014] de Santana Martins Rodgers, M. , Bavia, M. E. , Fonseca, E. O. L. , Cova, B. O. , Silva, M. M. N. , Carneiro, D. D. M. T. , Cardim, L. L. , & Malone, J. B. (2019). Ecological niche models for sand fly species and predicted distribution of *Lutzomyia longipalpis* (Diptera: Psychodidae) and visceral leishmaniasis in Bahia state. Brazil. Environmental Monitoring and Assessment, 191, 331 10.1007/s10661-019-7431-2 31254126

[ece36823-bib-0015] Dong, D. , Xu, X. T. , Zhou, Z. X. , He, Y. H. , Wang, C. Z. , Shi, F. Z. , & Gao, L. L. (2019). Niche dynamics of main populations of old‐tree communities in Jiuhua mountain senic area of Anhui province. Chinese Journal of Ecology, 38(5), 1292–1304. 10.13292/j.1000-4890.201905.023

[ece36823-bib-0016] Du, D. L. , Su, J. , & Liu, Y. C. (1997). Niche dynamics of *Castanopsisi fargesii* population. Chinese Journal of Applied Ecology, 8(2), 113–118. 10.13287/j.1001-9332.1997.0022

[ece36823-bib-0017] Gaston, K. J. , & Spicer, J. I. (2001). The relationship between range size and niche breadth: A test using five species of *Gammarus* (Amphipoda). Global Ecology and Biogeography, 10(2), 179–188. 10.1046/j.1466-822x.2001.00225.x

[ece36823-bib-0018] Gong, X. W. , & Lv, G. H. (2017). Species diversity and dominant species' niches of eremophyte communities of the Tugai forest in the Ebinur basin of Xinjiang. China. Biodiversity Science, 25(01), 34–45. 10.17520/biods.2016166

[ece36823-bib-0019] Grinnell, J. (1917). The niche‐relationships of the California thrasher. The Auk, 34(4), 427–433. 10.2307/4072271

[ece36823-bib-0020] Hu, Z. H. , Qian, H. Y. , & Yu, M. J. (2009). The niche of dominant species populations in *Castanopsis eyrei* forest in Gutian mountain national nature reserve. Acta Ecologica Sinica, 29(7), 3670–3677.

[ece36823-bib-0021] Hurlbert, S. H. (1978). The measurement of niche overlap and some relatives. Ecology, 59(1), 67–77. 10.2307/1936632

[ece36823-bib-0022] Iannella, M. , Cerasoli, F. , D’Alessandro, P. , Console, G. , & Biondi, M. (2018). Coupling GIS spatial analysis and ensemble niche modelling to investigate climate change‐related threats to the Sicilian pond turtle *Emys trinacris,* an endangered species from the Mediterranean. PeerJ, 6, e4969 10.7717/peerj.4969 29888141PMC5993018

[ece36823-bib-0023] Ingram, T. , Costa‐Pereira, R. , & Araujo, M. S. (2018). The dimensionality of individual niche variation. Ecology, 99(3), 536–549. 10.1002/ecy.2129 29282710

[ece36823-bib-0024] Jiang, Z. M. , Guan, W. , Xiong, Y. M. , Li, M. , Chen, Y. J. , & Liao, B. W. (2019). Interactive effects of intertidal elevation and light level on early growth of five mangrove species under *Sonneratia apetala* Buch. Hamplantation canopy: Turning monocultures to mixed forests. Forests, 10(2), 83 10.3390/f10020083

[ece36823-bib-0025] Lanszki, J. , Heltai, M. , Kövér, G. , & Zalewski, A. (2019). Non‐linear relationship between body size of terrestrial carnivores and their trophic niche breadth and overlap. Basic and Applied Ecology, 38, 36–46. 10.1016/j.baae.2019.06.004

[ece36823-bib-0026] Levins, R. (1968). Evolution in changing environments: Some theoretical explorations. Princeton University Press. ISBN 9780691080628.

[ece36823-bib-0027] Li, N. , Zeng, W. , Guo, Y. , Li, C. , Ma, C. , & Peng, Y. (2019). Nitrogen‐associated niche characteristics and bacterial community estimated by ^15^N‐DNA‐stable isotope probing in one‐stage partial nitritation/anammox process with different ammonium loading. Journal of Environmental Management, 247, 603–612. 10.1016/j.jenvman.2019.06.110 31276914

[ece36823-bib-0028] Liao, B. W. , Li, M. , Zheng, S. F. , Chen, Y. J. , & Zheng, X. R. (2003). Study on intraspecific and competition in exotic species *Sonneratia apetala* . Forest Research, 16(4), 418–422. 10.13275/j.cnki.lykxyj.2003.04.007

[ece36823-bib-0029] Lin, P. (1997). Mangrove ecosystem of China. Science Press. ISBN 9787030056924.

[ece36823-bib-0030] Liu, R. H. , Chang, B. , Rong, C. Y. , Jiang, Y. , Yang, R. A. , Liu, X. T. , Zeng, H. F. , & Fu, G. H. (2018). Niche of main woody plant populations of *Pterocarya stenoptera* community in riparian zone of Lijiang River. China. Chinese Journal of Applied Ecology, 29(12), 3917–3926. 10.13287/j.1001-9332.201812.001 30584717

[ece36823-bib-0031] López‐Alvarez, D. , Manzaneda, A. J. , Rey, P. J. , Giraldo, P. , Benavente, E. , Allainguillaume, J. , Mur, L. , Caicedo, A. L. , Hazen, S. P. , Breiman, A. , Ezrati, S. , & Catalán, P. (2015). Environmental niche variation and evolutionary diversification of the *Brachypodium distachyon* grass complex species in their native circum‐Mediterranean range. American Journal of Botany, 102(7), 1073–1088. 10.3732/ajb.1500128 26199365

[ece36823-bib-0032] Lou, Y. J. , Gao, C. Y. , Pan, Y. W. , Xue, Z. S. , Liu, Y. , Tang, Z. H. , Jiang, M. , Lu, X. G. , & Rydin, H. (2018). Niche modelling of marsh plants based on occurrence and abundance data. Science of the Total Environment, 616–617, 198–207. 10.1016/j.scitotenv.2017.10.300 29121575

[ece36823-bib-0033] Marinšek, A. , Čarni, A. , Šilc, U. , & Manthey, M. (2015). What makes a plant species specialist in mixed broad‐leaved deciduous forests? Plant Ecology, 216(10), 1469–1479. 10.1007/s11258-015-0527-z

[ece36823-bib-0034] Martínez, C. (2010). Trophic niche breadth and overlap of three egret species in a neotropical mangrove swamp. Waterbirds, 33(3), 285–292. 10.1675/063.033.0303

[ece36823-bib-0035] Mays, H. L. J. R. , Hung, C. M. , Shaner, P. J. , Denvir, J. , Justice, M. , Yang, S. F. , Roth, T. L. , Oehler, D. A. , Fan, J. , Rekulapally, S. , & Primerano, D. A. (2018). Genomic analysis of demographic history and ecological niche modeling in the endangered sumatran rhinoceros *Dicerorhinus sumatrensis* . Current Biology, 28(1), 70–76.e4. 10.1016/j.cub.2017.11.021 29249659PMC5894340

[ece36823-bib-0036] Mutshinda, C. M. , & O’Hara, R. B. (2011). Integrating the niche and neutral perspectives on community structure and dynamics. Oecologia, 166(1), 241–251. 10.1007/s00442-010-1831-x 21076983

[ece36823-bib-0037] Pagani‐Núñez, E. , Barnett, C. R. A. , & Senar, J. C. (2019). Age and sex differences in niche use at molt and its effect on plumage coloration characteristics in a bird. Current Zoology, 65(3), 251–260. 10.1093/cz/zoy062 31263483PMC6595419

[ece36823-bib-0038] Pianka, E. R. (1973). The structure of lizard communities. Annual Review of Ecology and Systematics, 4, 53–74. 10.2307/2096804

[ece36823-bib-0039] Ren, H. , Jian, S. G. , Lu, H. F. , Zhang, Q. M. , Shen, W. J. , Han, W. D. , Yin, Z. Y. , & Guo, Q. F. (2007). Restoration of mangrove plantations and colonisation by native species in Leizhou bay. South China. Ecological Research, 23(2), 401–407. 10.1007/s11284-007-0393-9

[ece36823-bib-0040] Rojo, C. , Mesquita‐Joanes, F. , Monrós, J. S. , Armengol, J. , Sasa, M. , Bonilla, F. , Rueda, R. , Benavent‐Corai, J. , Piculo, R. , & Segura, M. M. (2016). Hydrology affects environmental and spatial structuring of microalgal metacommunities in tropical pacific coast wetlands. PLoS One, 11(2), e0149505 10.1371/journal.pone.0149505 26900916PMC4762632

[ece36823-bib-0041] Sá‐oliveira, J. C. , Angelini, R. , & Isaac‐Nahum, V. J. (2014). Diet and niche breadth and overlap in fish communities within the area affected by an Amazonian reservoir (Amapá, Brazil). An Acad Bras Cienc, 86(1), 383–405. 10.1590/0001-3765201420130053 24676175

[ece36823-bib-0042] Schoener, T. W. (1968). The Anolis lizards of Bimini: Resource partitioning in a complex fauna. Ecology, 49, 704–726. 10.2307/1935534

[ece36823-bib-0043] Shannon, C. E. , & Weiner, W. (1949). The mathematical theory of communication: Unknown distance function. University of Illinois Press. ISBN 9780252725487.

[ece36823-bib-0044] Simpson, E. H. (1949). Measurement of diversity. Nature, 163, 688 10.1038/163688a0

[ece36823-bib-0045] Song, Y. C. (2001). Vegetation ecology. East China Normal University Press. ISBN 9787040461596.

[ece36823-bib-0046] Spies, T. A. , Franklin, J. F. , & Klopsch, M. (1990). Canopy gaps in Douglas‐fir forests of the cascade mountains. Canadian Journal of Forest Research, 20(5), 649–658. 10.1139/x90-087

[ece36823-bib-0047] Su, Z. Y. , Wu, D. R. , & Chen, B. G. (2003). Niche characteristics of dominant populations in natural forest in north Guangdong. Chinese Journal of Applied Ecology, 14(1), 25 10.13287/j.1001-9332.2003.0006 12722433

[ece36823-bib-0048] Sullivan, M. J. P. , Davy, A. J. , Grant, A. , & Mossman, H. L. (2018). Is saltmarsh restoration success constrained by matching natural environments or altered succession? A test using niche models. Journal of Applied Ecology, 55(3), 1207–1217. 10.1111/1365-2664.13033 29780171PMC5947831

[ece36823-bib-0049] Trivedi, C. , Reich, P. B. , Maestre, F. T. , Hu, H.‐W. , Singh, B. K. , & Delgado‐Baquerizo, M. (2019). Plant‐driven niche differentiation of ammonia‐oxidizing bacteria and archaea in global drylands. The ISME Journal, 13(11), 2727–2736. 10.1038/s41396-019-0465-1 31249390PMC6794256

[ece36823-bib-0050] Walker, B. (1995). Conserving biological diversity through ecosystem resilience. Conservation Biology, 9, 747–752. 10.1046/j.1523-1739.1995.09040747.x

[ece36823-bib-0051] Wang, B. S. , Li, M. G. , & Peng, S. L. (1995). Phytopopulology. Higher Education Press.

[ece36823-bib-0052] Winemiller, K. O. , Fitzgerald, D. B. , Bower, L. M. , & Pianka, E. R. (2015). Functional traits, convergent evolution, and periodic tables of niches. Ecology Letters, 18(8), 737–751. 10.1111/ele.12462 26096695PMC4744997

[ece36823-bib-0053] Zhang, J. T. (1995). Ecology of vegetation quantity. Science and Technology Press. ISBN 9787504613134.

[ece36823-bib-0054] Zuppinger‐Dingley, D. , Schmid, B. , Petermann, J. S. , Yadav, V. , Deyn, G. B. D. , & Flynn, D. F. B. (2014). Selection for niche differentiation in plant communities increases biodiversity effects. Nature, 515(7525), 108–111. 10.1038/nature13869 25317555

